The article "An Automated Toxicity Classification on Social Media Using LSTM and Word Embedding" was retracted in 2023. Reason: concerns about the peer review.

# An Automated Toxicity Classification on Social Media Using LSTM and Word Embedding

**DOI:** 10.1155/2022/8467349

**Published:** 2022-02-15

**Authors:** Ahmad Alsharef, Karan Aggarwal, Sonia, Deepika Koundal, Hashem Alyami, Darine Ameyed

**Affiliations:** ^1^Yogananda School of Artificial Intelligence, Computing and Data Science, Shoolini University, Solan, Himachal Pradesh 173229, India; ^2^Electronics and Communication Engineering Department, Maharishi Markandeshwar (Deemed to be University), Mullana, Ambala 133207, India; ^3^Department of Systemics, School of Computer Science, University of Petroleum & Energy Studies, Dehradun, India; ^4^Department of Computer Science, College of Computers and Information Technology, Taif University, P.O. Box 11099, Taif 21944, Saudi Arabia; ^5^System Engineering Department, Ecole de Technologie Supérieure, University of Quebec, Montreal, Canada

## Abstract

The automated identification of toxicity in texts is a crucial area in text analysis since the social media world is replete with unfiltered content that ranges from mildly abusive to downright hateful. Researchers have found an unintended bias and unfairness caused by training datasets, which caused an inaccurate classification of toxic words in context. In this paper, several approaches for locating toxicity in texts are assessed and presented aiming to enhance the overall quality of text classification. General unsupervised methods were used depending on the state-of-art models and external embeddings to improve the accuracy while relieving bias and enhancing F1-score. Suggested approaches used a combination of long short-term memory (LSTM) deep learning model with Glove word embeddings and LSTM with word embeddings generated by the Bidirectional Encoder Representations from Transformers (BERT), respectively. These models were trained and tested on large secondary qualitative data containing a large number of comments classified as toxic or not. Results found that acceptable accuracy of 94% and an F1-score of 0.89 were achieved using LSTM with BERT word embeddings in the binary classification of comments (toxic and nontoxic). A combination of LSTM and BERT performed better than both LSTM unaccompanied and LSTM with Glove word embedding. This paper tries to solve the problem of classifying comments with high accuracy by pertaining models with larger corpora of text (high-quality word embedding) rather than the training data solely.

## 1. Introduction

With the increased dependence on machine learning (ML) models for different purposes and tasks, researchers recognized the existence of unfairness in machine learning models as one of the most important challenges facing users of ML technologies, as most of these models are trained using human-generated data, which means human bias will emerge clearly in these models. In other words, ML models are biased as the humans who generated the data of training. Machine learning models' designers must take the initiative in recognizing and relieving these biases; otherwise, the models might propagate unfairness in classification [1]. This unintended bias in the models can also be a result of the demographics of the online users, the underlying or overt biases of those doing the labelling or the selection and sampling [2].

This work aims to improve the classification accuracy of toxicity in online chat forums, but the classification methods presented here can be applied to any other classification purpose. Toxicity is explained as anything that is insolent, uncivil, or excessive that would make someone want to leave a conversation. Machine learning models will usually learn the simplest associations to predict the corresponding labels of inputs, so any biases or incorrect associations in the training data can propagate unintended biased associations in the classification results. Trained models are known to have the ability to capture contextual dependencies. However, with insufficient data, the models might cause errors and become unable to identify the dependency model and become more probable to generalize, causing the false-positive bias in classification. Toxicity classification models specifically have been shown to capture biases that are common in society from society-generated training data and repeat these biases in classification results, for example, miss-associating frequently attacked identity groups, such as “Black” and “Muslim”, with toxicity in any context even in nontoxic contexts. The following sections will include a description of related works. Furthermore, on proposed models, a technique has been applied by embedding data to relieve the bias. Finally, metrics used for evaluating the classification accuracy in a model will demonstrate that the proposed techniques reduce bias while enhancing overall models' quality and accuracy.

## 2. Related Works

Prominent researchers have worked in the area of text analysis. They have analyzed the text and put several security features for its authentication [3, 4]. Authentic data can assist in reducing text toxicity, since not everyone reveals themselves while posting unwanted data.

Many other efforts have been put forward so far to solve the problem of classification in texts [5–11]. Various recent works have studies how concepts of fairness and unintended bias are applied to machine learning models. Researchers have proposed various metrics for the evaluation of fairness in models. Kleinberg et al. [12] and Friedler et al. [13], both groups of researchers, compared different fairness metrics. These works depended on the availability of demographic data to distinguish and relieve bias. Beutel et al. [14] presented a new mitigation technique that used adversarial training techniques and only required a small amount of deceptive labelled demographic data for training. Other works have been conducted on fairness for text classification tasks. Some researchers [15] analyzed different sentiment analysis techniques on the Turkish language with supervised and unsupervised ensemble models to explore the predictive efficiency of the term weighting schemes which is a process to compute and assign a numeric value to each term. The results indicated that supervised term weighting models can outperform unsupervised models in term weighting. Blodgett et al. [16], Hovy et al. [17], and Tatman [18] discussed the impact of using unfair models on real-world tasks but did not provide solutions to adjust this impact. Paryana et al. [19] have suggested intrusion detection techniques to catch such kinds of people. However, directly how it can be applied to the present problem has not been determined. Bolukbasi et al. [20], in 2016, demonstrated gender bias in word embeddings and provided a solution to counter it using fairer embeddings. Prominent authors [21] proposed an ensemble method for text sentiment analysis and classified it. It aggregates individual features obtained by different methods to obtain a crisp feature subset, and this proposed method outperformed the previous technique. Also, Onan [22] proposed an approach which uses TF_IDF glove embedding technique that gives better results in comparison to the conventional deep learning models in sentiment analysis.

Onan et al. [23] proposed a technique that contains a three-layer bidirectional LSTM network which showed a promising efficiency with a classification accuracy of 95.30%. Also, Onan [24] presented sentiment classification in MOOC reviews. In [25], researchers presented a machine learning-based approach to analyze sentiments with a corpus of 700 student reviews of higher educational institutions written in Turkish, and this machine learning-based approach achieved efficiency in analyzing the sentiments of these reviews.

Georgakopoulos et al. [26] compared convolutional neural networks (CNNs) against the traditional Bag-of-Words for text analysis where the frequency of each word is used as a feature for training combined with algorithms proven to be effective in text classification such as support vector machines (SVMs), Naïve Bayes (NB), K-nearest neighbours (KNNs), and linear discriminant analysis (LDA). They used the same as one of the datasets used in our experiments [27]. A CNN network pretrained with Word2Vec word embedding achieved the highest performance with respect to precision and recall and had the lowest false-positive ratio meaning that this CNNword2vec mistakenly predicted nontoxic comments as toxic the lowest number of times compared to the other models.

In [28], researchers presented an ensemble scheme based on depending on cuckoo search and k-means algorithms. The performance of the proposed model was compared to the conventional classification models and other ensemble models using 11 text benchmarks. The results indicated that the proposed classifier outperforms the conventional classification and ensemble learning model.

This paper adds to this growing effort of research intoxicity classification, an analysis of approaches to relieve bias in text classification tasks achieving high accuracy and F1-score which were the measures of classification as in [29]. Our proposed model used pretrained word embeddings to pertaining classification models instead of training them on the training dataset solely which causes vulnerability to bias.

## 3. Materials and Methods

This section should contain sufficient detail so that all procedures can be repeated. It may be divided into headed sections if several methods are described.

In this work, several text classifiers were built to identify toxicity in comments from public forums and social media websites. The performance of cache must be good to implement such kind of classifiers as suggested by Sonia et al. [30]. These classifiers were trained depending on two datasets and tested depending on one dataset.

The first training dataset [31] was of 1.8 million comments, labelled by human raters as toxic and nontoxic. The target column value measures the toxicity rate and determines whether the comment is toxic or not.

The second training dataset [27] was of 223,549 comments labelled in six categories of “toxic,” “severe toxic,” “insult,” “threat,” “obscene,” and “identity hate.”

The testing dataset [32] contained 97,321 entries labelled as approved meaning nontoxic or rejected meaning toxic.

The project focused on the effect of word embeddings on LSTM model binary classification accuracy. Given an input of a comment, it returns whether this comment is toxic or nontoxic. The metrics of measuring the classification accuracy were accuracy score and F1-score. The steps followed in the experimental work are illustrated in Figure 1.

The models applied in this work are illustrated in Table 1.

### 3.1. Analysis of the 1st Training Dataset

The first training dataset [31] was published by the Jigsaw unit of Google [33] throughout the competition of “Jigsaw Unintended Bias in Toxicity Classification” on the Kaggle community. Each comment in this dataset had a toxicity label (target). This attribute is a fractional value that represents the judgment of human raters who estimated how much toxicity is contained in a given comment. For classification accuracy evaluation, test set examples with (target ≥0.5) were considered as toxic, while other comments having target <0.5 were considered as nontoxic.  Table 2 is a tiny sample of these comments and their corresponding “target” value.

From Table 2, we observe that the first two comments are not toxic having target <0.5, whereas the third comment is toxic having target >0.5.

Terms affected by the false-positive bias usually occur in comments and are usually misclassified by NLP models as toxic even in nontoxic comments especially that the training data of models is usually human generated. The disproportionate number of toxic examples containing these terms in the training dataset can lead to overfitting in the classification model. For example, in this dataset, the word “gay” appears in only 3% of toxic comments and only 0.5% of the overall comments. Biased models can make overfitting such as always linking the word “gay” with toxicity which is not always correct, and it can come in a nontoxic context.

Visualization of data is reported in the next paragraphs.

We can see a relation between the target and certain categories of toxic words. The scatter charts illustrated in Figure 2 show the relationship between some of these categories and toxicity (target value).

The occurrence of comments holding these categories such as insult and identity attack increases its potential to be classified as toxic in the training dataset.

On the contrary, some words occurrence does not usually lead to toxicity. This is concluded from the scatter charts illustrated in Figure 3 which show the relation between some categories of comments and toxicity.

The occurrence of comments holding these words, such as black and Buddhist, does not usually increase its potential to be classified as toxic in the training dataset.

### 3.2. Analysis of the 2nd Training Dataset

The second training dataset [27] used in this work included 223,549 published by the Jigsaw unit of Google [33] throughout the “Toxic Comment Classification Challenge” on Kaggle. These user comments were labelled by human labellers within six labels: “toxic,” “severe toxic,” “insult,” “threat,” “obscene,” and “identity hate.” Some comments could be categorized into different labels at once. The dataset labels distribution is shown in Table 3.

Two lakh one thousand and eighty one comments were classified under the “clean” category matching none of the six categories constituting 89.9% of overall comments, whereas the other comments belonged to at least one of the other classes constituting 10.1% of overall comments. The comments collected were mostly written in English with some outliers of comments from different languages, e.g., in Arabic and Chinese. The comment was considered as “toxic” if it was classified under any of the six categories and as “nontoxic” otherwise (not categorized under any of the six categories).

### 3.3. Training Data Preprocessing

The text data preprocessing techniques followed before processing and modeling the data are as follows.

Punctuation removal: removing punctuation is a necessary step in cleaning the text data before performing analytics. In this work, all punctuation marks in all comments were removed.

Lemmatization: lemmatization is the process of grouping together the inflected forms of a word so they can be analyzed as a single term. In this work, lemmatization was performed for every comment.

Stop words' removal: stop words are words that do not contain any significance in a context. Usually, these words are filtered out from text blocks because they have unnecessary information such as the, be, are, and a.

### 3.4. Testing Dataset

The test dataset used for evaluation in this work was downloaded from the Kaggle competition of “Jigsaw Unintended Bias in Toxicity Classification” [32]. It contained 97321 entries labelled as approved (nontoxic) or rejected (toxic). A sample of the testing dataset is given in Table 4:

### 3.5. LSTM Model

Initially, LSTM [34, 35] was created where the information flows through cell states. In this way, LSTMs can selectively remember or forget information. This study worked on using LSTM and word embeddings for toxicity classification. The design of the LSTM neural networks used in this work is shown in Figure 4.

The designed fine-tuned LSTM of this work takes a sequence of words as an input.

A word embeddings' layer that provides a representation of words and their relative meanings was added. This embedding layer transforms encoded words into a vector representation.

Then, a spatial dropout layer that masks 10% of the word embeddings' layer output makes the neural network more robust and less vulnerable for overfitting.

Then, to process the resulted sequence, an LSTM layer with 128 units was used as well as another 10% dropout layer.

After all, a dense output layer was used to output the multilabel classification.

### 3.6. Word Embedding

Word embedding is a concept used for representing words for text analysis, generally in a form of a vector of real values that encodes the meaning of the word in such a way where the words that are closer in the vector space are expected to have related meanings [36]. Word embeddings can be obtained using different techniques where words from the vocabulary are mapped to vectors of real numbers. Each word is mapped to one vector.  Figure 5 illustrates the different types of word embeddings.

In this work, Glove static (context-independent) word embeddings and a contextualized word embeddings generated by BERT were used for pretraining the classification models before training them on the training datasets. The word embedding this work used is as follows.

Glove: it is a learning algorithm for calculating vector representations of words regardless of sentence context. Training in glove is performed on aggregated global word occurrence statistics from a large corpus [37, 38]. The Glove word embeddings this work used to pretrain the models are as follows:

Wikipedia 2014: 400 thousand word vectors trained on a largeWikipedia-2014 corpus [39].

Gigaword 5: Gigaword Fifth Edition archive of newswire text [40].

Twitter: 1.2 million word vectors trained on large Twitter corpora [4].

BERT: it is an encoder was proposed in a paper published by Google AI in 2018 [34, 41]. Its main innovation is to apply bidirectional training to the transformer, which is a well-known attention model in language modeling. Results predict that a bidirectionally trained language model can sense more deeply in context of language in comparison to the single directional language model. Bidirectional LSTM can also be trained on both sides that are left to right for detecting the next word of sentence and vice versa to find out the previous word. That means this will use both forward and backward LSTMs. However, none of the techniques considered both ways simultaneously like taken in BERT [19]. BERT also can generate various context-dependent word embeddings of a word dynamically informed by words around it [42].

## 4. Results and Discussion

The evaluation metrics used to evaluate the efficiency of models were accuracy and F1-score. The following paragraph will describe these metrics:

(i) Accuracy describes the accuracy achieved on the testing set. The formula for accuracy is
  (1) $$\begin{array}{c} \text{Accuracy}=\frac{\text{Number of correct predictions}}{\text{Total number of predictions}}. \end{array}$$
(ii) Precision is defined as the ratio of correctly predicted positive observations to the total predicted positive observations. The formula for precision is
  (2) $$\begin{array}{c} \text{Precision}=\frac{\text{TP}}{\text{TP}+\text{FP}}. \end{array}$$
(iii) Recall is defined as the proportion of correctly identified positives. The formula for recall is
  (3) $$\begin{array}{c} \text{Recall}=\frac{\text{TP}}{\text{TP}+\text{FN}}. \end{array}$$
(iv) F1-score is the harmonic mean of precision and recall. The formula for F1-score is
  (4) $$\begin{array}{c} \text{F}1=\frac{2}{{\text{precision}}^{-1}+{\text{recall}}^{-1}}\\ =2\cdot \frac{\text{precesion}.\text{recall}}{\text{precesion}+\text{recall}}\\ =\frac{\text{TP}}{\text{TP}+\left(1/2\right)\left(\text{FP}+\text{FN}\right)}. \end{array}$$

The experiments applied the LSTM model by pertaining it with different word embeddings each time. The LSTM model itself is known for its memory that can keep long sequences of words and its suitability for word classification. After adding the Glove word-embedding layer and applying the LSTM model, we obtained a high accuracy of 93% and a high F1-score of 0.84 on the previously mentioned training and testing datasets. However, in LSTM, according to Singh [19], the language models built on word embeddings do not accurately capture the nuances and meanings of the sentences. This made the added word embeddings not highly effective for language modeling. Using bidirectional word embeddings solved the problem where combining LSTM with BERT and applying the same settings as in the previous model gave a higher classification accuracy of 94% and a higherF1-score of 0.89, in classifying toxic comments, on the previously mentioned training and testing datasets. The summary of the results are represented in Table 5.

From the results, we could find that using word embeddings could improve the efficiency of classification. Words embedding generated by the BERT model was proved to be more efficient than static Glove word embeddings when used with LSTM since it trains in both directions allowing higher efficiency, and because BERT analyzes every sentence with no specific direction, it does a better job at understanding the meaning of homonyms than previous NLP methodologies, such as Glove embedding methods.

Word embeddings trained on a large corpus such as Glove trained on Wikipedia, Gigword, and Twitter were also found effective to enhance the accuracy of classification but less effective than BERT (in classifying toxicity in text documents).

## 5. Conclusions

Many former research works have recognized unfairness in ML models for toxicity classification causing inaccurate classification as a concern to relieve. This can be observed obviously in toxicity classification in public talk pages and online discussion forums. In this paper, various machine learning and natural language processing models for toxicity classification were proposed, implemented, and illustrated. It was found that many errors in toxicity identification occur due to the lack of consistent quality of data. By adding word embeddings, the accuracy of classification increased notably. Finally, an accuracy of 94% and an F1-score of 0.89 were achieved using a hybrid BERT and LSTM classification model. This work can be further extended by exploring the potential of subword embeddings [43] which can further enhance the accuracy of classification. A more robust model can be developed by applying AutoNLP and AutoML techniques on the same datasets where in order to obtain better results and accurate classifications these techniques automatically find the models that fit data the best.

## Figures and Tables

**Figure 1:** Experimental workflow.

**Figure 2:** The relation between some features of comments and toxicity in the 1^st^ training dataset.

**Figure 3:** The relation between some features of comments and toxicity.

**Figure 4:** LSTM model layers' design.

**Figure 5:** Word embedding types.

**Table 1:** Classification models of this work.

Experiment 1		Experiment 2	
Neural network	Word embedding	Neural network	Word embedding
LSTM	Glove	LSTM	BERT

**Table 2:** Training dataset 1 sample.

Comment_text	Target
This is so cool. It's like, “would you want your mother to read this??'”	0
Thank you!! This would make my life a lot less anxiety-inducing.	0
Haha, you guys are a bunch of losers.	0.8936

**Table 3:** Label distribution of the 2^nd^ training dataset.

Class	No. of occurrences
Clean	201,081
Toxic	21,384
Obscene	12,140
Insult	11,304
Identity hate	2,117
Severe toxic	1,962
Threat	689

**Table 4:** Testing dataset sample.

Comment_text	Rating
Sorry, you missed high school. Eisenhower sent troops to Vietnam after the French withdrew in 1954	Approved
Our oils read; President IS taking different tactics to deal with a corrupt malignant, hypocritical ….	Rejected
Why would 90% of articles print fake news to discredit Trump? Where are you getting your new” …	Approved

**Table 5:** Accuracy and F1-score of LSTM with different word embeddings in classifying toxic words.

	Accuracy (%)	F1-score
**LSTM** **+** **Glove**	93	0.841
**LSTM** **+** **BERT**	94	0.894

## Data Availability

The data presented in this study are openly available in Kaggle competition of “Jigsaw Unintended Bias in Toxicity Classification.”
